RETRACTED

# The Role of LINC00284 in the Development of Thyroid Cancer *via* Its Regulation of the MicroRNA-30d-5p-Mediated ADAM12/Notch Axis

**DOI:** 10.3389/fonc.2021.643039

**Published:** 2021-08-18

**Authors:** Chunmei Hu, Zhichen Kang, Lixin Guo, Fuling Qu, Rongfeng Qu

**Affiliations:** ^1^Department of Hematology and Oncology, The Second Hospital of Jilin University, Changchun, China; ^2^Rehabilitation Department, The Second Hospital of Jilin University, Changchun, China

**Keywords:** Thyroid cancer, long non-coding RNA, LINC00284, MicroRNA-30d-5p, A disintegrin and metalloproteinase 12, Notch signaling pathway, self-renewal

## Abstract

Thyroid cancer is a commonly diagnosed endocrine malignancy with increasing incidence worldwide. Long noncoding RNAs (lncRNAs) are known to function in the invasion and metastasis of thyroid cancer. According to the GSE66783 microarray dataset, long intergenic nonprotein coding RNA 284 (LINC00284) is aberrantly upregulated in thyroid cancer tissues. However, information regarding the specific role of LINC00284 in thyroid cancer remains elusive. Therefore, the current study set out to determine the role of LINC00284 in the development of thyroid cancer, along with an investigation of the underlying molecular mechanism. In parallel with the microarray data from GSE66783, LINC00284 was observed to be expressed at high levels in thyroid cancer cell lines. Moreover, loss-of-function experiments revealed that the downregulation of LINC00284 reduced aldehyde dehydrogenase (ALDH) activity and thyroid cancer cell proliferation, colony formation, and invasiveness, which promoted cell apoptosis. Mechanistically, using dual-luciferase reporter, RNA pull-down, and RNA immunoprecipitation (RIP) assays, LINC00284 was identified to competitively bind to microRNA-30d-5p (miR-30d-5p), which was observed to be expressed at low levels in thyroid cancer tissues and cells and directly targets the oncogene a disintegrin and metalloproteinase 12 (ADAM12). Overexpression of miR-30d-5p exerted tumor-suppressive effects on the malignant activity of thyroid cancer cells, changes that were reversed by LINC00284 overexpression or ADAM12 overexpression. Furthermore, LINC00284 activated the Notch signaling pathway by competitively binding to miR-30d-5p and increasing the expression of ADAM12. Finally, by performing *in vivo* experiments, we found that LINC00284 silencing or miR-30d-5p overexpression suppressed the tumorigenic ability of thyroid cancer cells and that overexpression of miR-30d-5p inhibited the LINC00284-induced tumorigenesis of thyroid cancer cells. Collectively, our findings indicate that LINC00284 competitively binds to miR-30d-5p and activates the ADAM12-dependent Notch signaling pathway, thereby promoting the development of thyroid cancer.

RETRACTED

## Introduction

Thyroid cancer is one of the most common endocrine malignancies worldwide, with the incidence increasing steadily in the last few decades (1). Furthermore, thyroid cancer accounts for 1% of all cancers, is primarily diagnosed in middle-aged people, and results in higher morbidity in women, while its poor prognosis is mainly attributed to an inadequate understanding of its regulatory networks (2). Thyroid cancer is a heterogeneous group of cancers that are classified into several subtypes, including papillary thyroid cancer (PTC) and follicular thyroid cancer (FTC) (3). Moreover, numerous factors, such as genetic changes, growth factors, and radiation, are implicated in the development of PTC, with radiation exposure being the most well-known risk factor (4), while age, tumor size, and histological parameters, including lymph node invasion and distant metastasis, are also associated with the prognosis of PTC (5). Recent advancements in the field of medical research have shown that numerous long noncoding RNAs (lncRNAs) are dysregulated in PTC and function as diagnostic and prognostic biomarkers of this cancer, indicating the therapeutic potential of lncRNAs (6, 7).

LncRNAs serve as important factors contributing to various biological processes, including transcriptional regulation and cell growth, and are thus involved in the carcinogenesis and aggressiveness of PTC (8). As reported previously, long intergenic nonprotein coding RNA 460 (LINC00460) promotes the progression of papillary thyroid cancer by regulating the LINC00460/miR-485-5p/Raf1 axis (9). Moreover, LINC00284 was previously reported to function as a tumor-promoting lncRNA in ovarian cancer by enhancing the proliferation, migration, invasion, and tumorigenic ability of ovarian cancer cells (10). Additionally, increasing data suggest that several lncRNAs function as competing endogenous RNAs (ceRNAs) for shared miRNAs to regulate the distribution of miRNAs on the targets at a posttranscriptional level (11, 12). Moreover, abnormally expressed miRNAs are implicated in the pathogenesis of numerous cancers, including thyroid cancer (13). For example, miR-145 was reported as a diagnostic biomarker for thyroid cancer (14). Additionally, miR-30d was shown to confer an antitumor effect on anaplastic thyroid carcinoma (15). In addition, a recent study also highlighted the tumor-suppressive effect of miR-30d-5p on prostate cancer (16). Initial prediction results from the miRDB website in the current study indicated that ADAM12 might be a target gene of miR-30d-5p. A disintegrin and metalloproteinase 12 (ADAM12), a metalloproteinase of the zinc protease superfamily, is known to be involved in carcinogenesis through diverse mechanisms (17). Interestingly, a hypoxia-induced increase in the activity of ADAM12 was previously found to lead to cancer cell invasion through a Notch signaling-dependent mechanism (18). Based on the aforementioned literature, we speculated that LINC00284 and miR-30d-5p may play pivotal roles in thyroid cancer through regulatory effects on ADAM12 and the Notch signaling pathway. Therefore, the current study aimed to identify the effect of LINC00284 on thyroid cancer and the associated regulatory network.

RETRACTED

## Methods

### Ethics Statement

All experimental procedures involving animals were performed in strict accordance with the laboratory animal care and usage guidelines issued by the US National Institutes of Health (NIH). Optimal measures were taken to minimize animal suffering.

### Bioinformatics Analysis

The GSE66783 dataset, including five PTC samples and matched paracancerous tissue samples, was obtained from the Gene Expression Omnibus (GEO) database to validate the expression of LINC00284 in thyroid cancer samples (19). Then, the Gene Expression Profiling Interactive Analysis (GEPIA) database (http://gepia2.cancer-pku.cn/#index) was used to identify the expression of LINC00284 in thyroid cancer samples and normal samples collected in The Cancer Genome Atlas (TCGA) and the Genotype-Tissue Expression (GTEx) databases. Next, the intracellular localization of LINC00284 was predicted using the bioinformatics website lncLocator. The interactions between LINC00284 and miRNAs were determined using the miRDB website (http://www.mirdb.org/mirdb/policy.html). The potential target gene of miR-30d-5p, ADAM12, was predicted through a bioinformatics analysis (http://www.microrna.org). Finally, using the starBase online database (starbase.sysu.edu.cn/), the pattern of ADAM12 expression in thyroid cancer samples in the TCGA database was identified, followed by a correlation analysis of miR-30d-5p and ADAM12 expression in thyroid cancer.

### Cell Culture

A normal thyroid epithelial cell line (HT-ori3) and five thyroid cancer cell lines (SW1736, FTC133, WRO82, HTh74, and C643) were acquired from the American Type Culture Collection (Manassas, VA, USA). The aforementioned cells were cultured in Dulbecco’s modified Eagle’s medium (DMEM) (Gibco, Carlsbad, CA, USA) supplemented with a combination of 10% fetal bovine serum (FBS), 1% minimum essential medium (MEM), 100 U/mL penicillin, and 100 mg/L streptomycin under saturated conditions of 37°C and 5% CO_2_. Upon attaining 80%-90% cell confluence, the third generation of cells was subcultured by treatment with trypsin to harvest the monolayer cells and subsequent inoculation in a 24-well plate.

RETRACTED

### Plasmid Construction and Cell Grouping and Transfection

According to the identified sequences of LINC00284, miR-30d-5p, and ADAM12 obtained from the National Center for Biotechnology Information (NCBI), a negative control (NC) empty plasmid, short hairpin RNA targeting LINC00284 (sh-LINC00284), LINC00284 overexpression plasmid (oe-LINC00284), mimic-NC, miR-30d-5p mimic, and oe-ADAM12 plasmids were designed and constructed by Shanghai Sangon Biotechnology Co. Ltd. (Shanghai, China).

For cell grouping, the third generation of cultured thyroid cancer cell lines was trypsinized, seeded into 24-well plates, and cultured into a monolayer. The thyroid cancer cell line HTh74 was treated with sh-NC, sh-LINC00284, sh-LINC00284 + DMSO, or sh-LINC00284 + TBHQ. Another cell line, C643, was untransfected or transfected with the miR-30d-5p mimic, oe-LINC00284, oe-ADAM12, and their corresponding controls (mimic-NC or oe-NC) individually or in combination.

Cell transfection was executed using Lipofectamine 2000 (Invitrogen, Carlsbad, CA, USA) in strict accordance with the provided instructions. Specifically, 2×10^5^ HTh74 and C643 cells were seeded in each well of a 6-well plate. After the cells adhered to the plates and 12 h before transfection, the culture media were replaced with a fresh culture medium without penicillin-streptomycin. Next, 100 μL of Lipofectamine 2000 and 4 μg of plasmid were separately diluted in 250 μL of Opti-MEM, mixed and incubated at room temperature for 5 min followed by mixing the two preparations and an incubation at room temperature for 20 min. Then, the aforementioned transfection preparation was added to 6-well plates containing 1.5 mL of Opti-MEM, mixed and cultured in an incubator at 37°C with 5% CO_2_. The culture media were replaced with a complete medium 6 h after transfection. Cells were seeded in a G418 (1000-2000 μg/mL) medium at 48 h after transfection and cultured for 4 weeks with a replacement of the culture medium every 3-5 days to screen stably transfected cell lines. The target sequence of sh-LINC00284 was 5’-GGTTCTATGCTTGCTGTAATT-3’, and the sequence of the miR-30d-5p mimic was 5’-UGUAAACAUCCCCGACUGGAAG-3’.

### RNA-Fluorescence *In Situ* Hybridization (RNA-FISH)

The cytoplasm was isolated from the nucleus to identify the sublocalization of LINC00284. Transfected cells were treated with trypsin, centrifuged for 5 min, and resuspended in cold phosphate-buffered saline (PBS). After transfer of the cell suspension into a 1.5 mL Eppendorf tube, cells were centrifuged again for 2-3 min to eliminate the supernatant. The clean cells were fully incorporated with precooled ceruloplasmin (CER) I at the maximal rotation speed for 15 s and incubated on ice for 10 min for lysis, followed by the addition of precooled CER II under identical mixing conditions (at the maximal rotation speed) for 5 s. After an incubation on ice for 1 min, the cells were centrifuged for 5 min at 4°C.

RETRACTED

The obtained supernatant containing the cytoplasm was transferred to a new centrifuge tube and stored at -80°C for preservation, while the pellet was rinsed with PBS three times, and the precipitated cells were mixed with precooled nucleotide excision repair (NER) solution for 15 s at maximum speed. After a regimen of 40 min of incubation on ice, the cell-NER mixture was rotated for 15 s every 10 min and then centrifuged for 10 min at 4°C, after which the supernatant containing the nuclei was transferred into a new EP tube and stored at -80°C for preservation. Reverse transcription quantitative polymerase chain reaction (RT-qPCR) was performed to determine the location of LINC00284 in the cytoplasm and the nucleus (the primer sequences used in this study are listed in **Supplementary Table 1**).

Before the *in situ* hybridization experiment, the preparation was conducted on the first day (all reagents and instruments were RNase-free and operated at room temperature), including slide preparation and prehybridization. The slide was initially dried at 50°C for 15-30 min and then fixed with diethyl pyrocarbonate (DEPC)-4% polyfluoroalkoxy (PFA) for 20 min, followed by a rinse with 1 × DEPC-PBS A and then with 1 × DEPC-PBS B for 5 min. Subsequently, the slide was treated with proteinase K for 10 min and fixed again with DEPC-4% PFA for 10 min after a rinse with 1 × DEPC-PBS B. The slide was rinsed again with 1 × DEPC-PBS A and then with 1 × DEPC-PBS B for 5 min to eliminate the fixation solution prior to acetoxylation. Acetoxylation was conducted by incubating the slide with 0.1 M RNase-free triethylamine (TEA) at room temperature for 10 min, followed by sequential rinses with 1 × DEPC-PBS B and 1 × DEPC-PBS C for 5 min. Prehybridization was conducted with 200 μL of the prehybridization solution at room temperature for 1 h. Meanwhile, the RNA probes (0.1-0.2 ng/μL) (sequence: 5’-CCAGAUAUUUUACUUUUAAAUGUUUAC-3’) were prepared by denaturation in the prehybridization solution at 85°C for 5 min and placed on ice quickly.

When both the slide and RNA probes were ready, hybridization was conducted by adding the RNA probe to the slides and an incubation for 14 h at 65°C. On the second day, the slices were rinsed with preheated 0.2 × saline sodium citrate (SSC) A, B, and C at 65°C for three times (20 min each) and then with 0.2 × SSC D for 5 min, followed by two rinses with Buffer B 1 (5 min each). Afterwards, the slide was blocked with Buffer B 2 at room temperature for 1 h and then incubated with the anti-digoxin (DIG)-AP Fab antibody diluted with Buffer B 2 (1:5000) at 4°C overnight. On the third day, the slides were rinsed again three times with Buffer B 1 (20 min each), equilibrated twice with Buffer B 3 (5-10 min each), and finally stained with 5-bromo-4-chloro-3-indolyl phosphate (BCIP)/nitroblue tetrazolium (NBT) for 3-24 h in the dark, after which the coloration was terminated using ddH_2_O.

RETRACTED

### Dual-Luciferase Reporter Assay

A dual-luciferase reporter assay was conducted to identify the competitive binding of LINC00284 to miR-30d-5p. The total RNA content was extracted from HTh74 and C643 cells, and the LINC00284 wild-type and mutant primers (synthesized by Shanghai Sangon Biotechnology Co., Ltd., Shanghai, China) were amplified and cloned into the pmirGLO luciferase reporter vector (Promega, Madison, WI, USA) at the Pme I and Xba I restriction sites to conduct the dual luciferase reporter assay. Ligase IV was used to connect the amplified target gene and digested evector to construct LINC00284-Wt (wild type, 5’-UCCAGAUAUUUUACUUUUAAAUGUUUAC-3’) and LINC00284-Mut (mutant type, 5’-AGGUCAUAUUUUACUUUUAAUACAAAUG-3’) plasmids, which were transformed into *Escherichia coli*.

After polymerase chain reaction (PCR) to screen the positive clones containing the target plasmid, the product was sequenced. Next, 293T cells (American Type Culture Collection) were cotransfected with LINC00284-Wt and miR-30d-5p mimic plasmids, LINC00284-Mut and miR-30d-5p mimic plasmids, LINC00284-Wt and miR-30d-5p mimic-NC plasmids, or LINC00284-Mut plasmid and miR-30d-5p mimic-NC plasmids. Transfection was conducted using Lipofectamine 2000 (Invitrogen) according to the instructions provided. Six hours after transfection, the cells were incubated with a fresh medium for 24 h and then collected. The luciferase activity was detected with a dual-luciferase reporter assay kit (Promega) and a microplate reader (MK3, Thermo Fisher Scientific, San Jose, CA, USA) at 560 nm. The experiment was conducted three times to obtain the average value.

The relationship between miR-30d-5p and ADAM12 was validated by performing a dual-luciferase reporter assay. Specifically, the wild-type ADAM12 luciferase reporter plasmid (ADAM12-Wt) containing the wild-type ADAM12 sequence (5’-CCCCUCGCCACUGAUGUUUACU-3’) and the mutant ADAM12 luciferase reporter plasmid (ADAM12-Mut) containing the mutant ADAM12 sequence (5’-CCCGACUCAACUCUACAAAGGAUU-3’) were provided by GeneChem (Shanghai, China). 293T cells were cotransfected with ADAM12-Wt/ADAM12-Mut and miR-30d-5p mimic or miR-30d-5p mimic-NC. Transfection was conducted using Lipofectamine 2000 (Invitrogen) according to the instructions provided with the kit. Six hours after transfection, the culture medium was replaced, and the cells were collected after 24 h of incubation. The luciferase activity was detected at 560 nm using a dual-luciferase reporter assay kit (Promega) and a microplate reader (MK3, Thermo Fisher Scientific).

RETRACTED

### RNA Pull-Down and RNA Immunoprecipitation (RIP) Assays

The extracted total RNA for the dual luciferase activity experiment was also used here for transcription with an AmpliScribe T7-Flash Biotin-RNA Transcription Kit (Epicenter Technologies Corp., Madison, WI, USA) *in vitro*. The extracted RNA was first purified with an RNeasy Plus Mini Kit (Qiagen, Hilden, Germany) and DNase I (Qiagen). Subsequently, the purified RNA was biotin-labeled with Biotin RNA Labeling Mix (Ambion, Austin, TX, USA), and the biotin-labeled RNA was heated with an RNA structure buffer (10 mM Tris, pH 7.0, 0.1 M KCl and 10 mM MgCl_2_) at 90°C for 2 min, followed by an incubation on ice for 2 min and an incubation at ambient temperature for 20 min to form suitable secondary structures. Next, RNA was mixed with the total protein content of all the cells extracted above and incubated for 1 h, followed by an incubation with streptavidin-coated magnetic beads (Streptavidin Mag Sepharose, GE Healthcare, Chicago, Illinois, USA) for 1 h. Following rinses with ddH_2_O, the final RNA pull-down complex was collected for RT-qPCR. The primer sequences used in this study are listed in **Supplementary Table 1**.

The binding of LINC00284 to the AGO2 protein was detected using a RIP kit (Millipore Corp., Bedford, MA, USA). Cells were incubated with lysis buffer and enzyme inhibitors (1111111, Roche, Beijing Jiamei Biotech Co., Ltd., Beijing, China) for 5 min in an ice bath. Next, the supernatant was obtained after centrifugation at 14,000 rpm at 4°C for 10 min. One-third of the cell extract was removed as input, and the remaining two-thirds were incubated with 5 μg of AGO2 antibody (ab32381, dilution ratio of 1:50, Abcam, Cambridge, UK) for coprecipitation. Following homogenization for 30 min, IgG (ab109489, dilution ratio of 1:100, Abcam) and magnetic beads were resuspended in 100 μL of RIP washing buffer. After washing, the magnetic bead-antibody complexes were resuspended in 900 μL of RIP washing buffer and incubated with 100 μL of cell extract at 4°C overnight. The sample of the coprecipitation reaction system was placed on a magnetic stand to collect the magnetic bead-protein complexes. RNA was extracted from coprecipitation reaction system samples and the input after digestion, and the expression patterns of LINC00284 were detected using RT-qPCR. The primer sequences used in the present study are listed in **Supplementary Table 1**. The experiment was repeated three times to obtain the mean value.

RETRACTED

### Determination of Aldehyde Dehydrogenase Activity

After a 24-h transfection period, the cells were resuspended in ALDEFLUOER buffer to adjust the cell density to 1 × 10^6^ cells/mL. The activity of aldehyde dehydrogenase (ALDH) in each group was then detected according to the instructions of the ALDEFLUOER kit (STEMCELL Technologies, Inc., Vancouver, British Columbia, Canada). The detailed procedures are described below. Cells were incubated with 15 μmol/L ALDH-specific inhibitor diethylaminoazobenzene (DEAB) and 0.15 μmol/L ALDH substrate at 37°C for 25 min, followed by the detection of ALDH activity using a flow cytometer (Becton, Dickinson and Company, NJ, USA). The experiment was repeated three times to obtain the mean value.

### 3-(4,5-Dimethyl-2-Thiazolyl)-2,5-Diphenyl-2-H-Tetrazolium Bromide (MTT) Assay

The transfected cells were reacted with 20 μL of MTT (5 mg/mL, Sigma Chemical Co., St. Louis, MO, USA) at 0, 12, 24, 48, and 72 h after transfection. The cells were further cultured for 4 h in the dark. Next, the cells were treated with 150 μL of dimethyl sulfoxide (DMSO) for 10 min. An enzyme-linked immunometric meter (DG5031, Ke Huai Instrument Co., Ltd., Shanghai, China) was then used to detect the optical density value at an absorbance wavelength of 490 nm.

### Flow Cytometry

Twenty-four hours after transfection, the cells were treated with trypsin lacking ethylenediamine tetraacetic acid (EDTA) and centrifuged at 1118 × g for 5 min. The trypsin-treated cells were then rinsed with PBS twice and centrifuged. Next, the pellets were fixed with 3 mL of 70% precooled ethanol and then incubated overnight at 4°C. On the next day, the pellets were centrifuged and mixed with 0.5 mg/mL propidium iodide (PI) staining solution. After staining, the cells were filtered with a cell filter for PI detection with a flow cytometer (FACSCalibur, BD Company) at a wavelength greater than 575 nm to detect cell apoptosis.

For the determination of the cell apoptosis rate, cells were first cultured in a humidified incubator at 37°C with 5% CO_2_ for 48 h and stained with an Annexin V-fluorescein isothiocyanate (FITC)/PI double staining kit (556547, Shanghai Shuojia Bio Technology Co., Ltd., Shanghai, China). Briefly, the cells were stained with 5 µL of Annexin V-FITC for 15 min and 5 µL propidium iodide (PI) for 5 min, followed by detection using a flow cytometer (Cube6, Partec, Germany). FITC was detected at 530 nm, and PI was detected at wavelengths greater than 575 nm with an excitation wavelength of 480 nm.

RETRACTED

### Clone Formation Assay

Twenty-four hours after transfection, cells were detached with 0.25% trypsin and prepared as a single-cell suspension. Next, the cell suspension (1 × 10^4^ cells/mL) was cultured for 2 days in a 6-well plate. When cell clones were visible to the naked eye, the culture was terminated, and the supernatant was discarded, followed by two rinses with PBS and fixation with 3.7% methanol for 10 min. After staining with 0.1% crystal violet for 10-30 min, the cells were washed with running water and dried at room temperature. Finally, the number of clones containing more than 50 cells was counted under a low-power microscope.

### Cell Sphere Formation Assay

Twenty-four hours after transfection, the cells were incubated in a 96-well low-adhesion culture plate at a density of 200 cells/well with serum-free DMEM/F-12 containing B27 (1:50, Life Technologies, Carlsbad, CA, USA), basic fibroblast growth factor (20 ng/mL), and epidermal growth factor (20 ng/mL). Finally, the number of cell spheres (diameter > 50 μm) formed within 7 day was counted.

### Transwell Assay

Forty-eight hours after transfection, Matrigel (356234, BD Company, Franklin Lakes, NJ, USA) was incubated at 4°C overnight. After culture with a serum-free medium, the cell suspension (1 × 10^5^ cells/mL) was seeded into the apical chamber. Simultaneously, a medium containing 10% FBS was incubated in the basolateral chamber at 37°C for 24 h. The Transwell chamber was then rinsed with PBS twice for 5 min each and fixed with 5% glutaraldehyde at 4°C. Next, the Transwell chamber was stained with 0.1% crystal violet for 30 min and rinsed with PBS twice for 5 min each, followed by observation under a microscope. The number of cells passing through Matrigel was used as an index to evaluate the invasive ability.

### RT-qPCR

Total RNA was extracted using a TRIzol reagent (Takara Inc., Dalian, China). The purity and concentration of RNA were measured using a NanoDrop ND-1000 instrument (NanoDrop Technologies, San Francisco, CA, USA). The obtained RNA was reverse-transcribed into cDNAs with a PrimeScript RT reagent kit (Takara Co., Ltd, Dalian, China). U6 was used as an internal reference for miR-30d-5p, and real-time qPCR was performed to determine the relative miR-30d-5p expression patterns using a QuantiTect SYBR Green PCR kit. The reaction with a total volume of 20 μl contained 1 μl of cDNA templates, 0.4 μl of the forward primer, 0.4 μL of the reverse primer, 2 μL of 10 × miScript Universal Primer, 10 μL of 2 × QuantiTect SYBR Green PCR Master Mix and 6.2 μL of RNase-free ddH_2_O. Glyceraldehyde-3-phosphate dehydrogenase (GAPDH) was used as an internal reference for other genes, and a SYBR Premix Ex Taq II Kit (Takara, Tokyo, Japan) was applied to determine their expression patterns. A reaction system with a total volume of 20 μL contained 1 μL of cDNA templates, 0.4 μL of the forward primer, 0.4 μL of the reverse primer, 10 μl of SYBR Premix Ex Taq, 0.4 μL of ROX (50 ×) and 7.8 μL of ddH_2_O. All primers used in this experiment are listed in **Supplementary Table 1**. All RT-qPCR experiments were performed using an ABI7500 quantitative PCR instrument (Applied Biosystems, Foster City, CA, USA). The 2^-ΔΔCt^ method was applied to calculate the relative expression.

RETRACTED

### Western Blot Analysis

Seventy-two hours after transfection, the total cell protein content was extracted with radioimmunoprecipitation assay (RIPA) buffer containing protease inhibitors. The concentration of each protein sample was measured with bicinchoninic acid kits (Pierce, Rockford, IL, USA). Subsequently, 12.5% sodium dodecyl sulfate separation gel and concentration gel were prepared for protein separation by electrophoresis. The separated proteins were transferred to a polyvinylidene fluoride membrane, which was then blocked with 5% skim milk at 4°C overnight. On the next day, the membrane was incubated with the following diluted primary antibodies at 4°C overnight: rabbit anti-human Notch1 (dilution ratio of 1:800, ab65297), HES1 (dilution ratio of 1:200-2000, ab71559), and rabbit anti-human ADAM12 (dilution ratio of 1:100, ab39155). The membrane was then rinsed with PBS three times at room temperature for 5 min each and incubated with a goat anti-rabbit IgG secondary antibody (dilution ratio of 1:2000-20,000, ab6721) labeled with horseradish peroxidase at 37°C for 1 h. After development with enhanced chemiluminescence reagents (Pierce, Waltham, MA, USA), the protein bands were visualized. GAPDH (dilution ratio of 1:2500, ab9485) was used as the internal control, and the ratio of the gray value of the target band to the GAPDH band was calculated as the relative protein level. All the abovementioned antibodies were purchased from Abcam (Cambridge, UK).

### Tumorigenicity Assay in Nude Mice

Thirty female BALB/c mice (age 4 weeks old) were used for the experiment, with five mice in each group. The mice were provided free access to ordinary feed and water at room temperature with 50%-60% humidity, good ventilation, and a light/dark cycle of 12 h:12 h. Cells were stably infected with lentiviruses expressing oe-NC, oe-LINC00284, LV-NC, LV-miR-30d-5p, oe-LINC00284 + LV-NC, or oe-LINC00284 + LV-miR-30d-5p. The aforementioned lentiviruses were purchased from Wosunbio Co., Ltd. (Tanjin, China).

RETRACTED

Twenty-four hours after transfection, the cells were trypsinized, rinsed with PBS twice, and then suspended in serum-free RPMI 1640 medium. A total of 1.5 × 10^6^ cells were suspended in 0.1 mL of serum-free DMEM and mixed with 0.1 mL of extracellular matrix (ECM) gel. The cell-DMEM-ECM mixture was subcutaneously injected into the back of the nude mouse, and an equal number of cells were injected into the same site after 3 days. After injection, tumor formation was observed every 2 days, and the tumor volume was measured using Vernier calipers. At 4 weeks after the tumor formed, the nude mice were euthanized, and the tumor specimens were extracted to measure the weight and volume.

### Statistical Analysis

Statistical analyses were performed using SPSS 21.0 software (IBM Corp. Armonk, NY). Measurement data are presented as means ± standard deviations. Comparisons between two groups were analyzed using unpaired *t*-tests, while comparisons among multiple groups were analyzed using one-way analysis of variance (ANOVA) with Tukey’s *post hoc* test. Data collected at different time points were analyzed using repeated-measures ANOVA with Tukey’s *post hoc* test. A *p* value < 0.05 was regarded as statistically significant.

## Results

### LINC00284 Is Expressed at High Levels and miR-30d-5p Is Expressed at Low Levels in Thyroid Cancer Tissues and Cells

First, a differential expression analysis of microarray data in the GSE66783 dataset revealed that LINC00284 was expressed at high levels in thyroid cancer (**Figure 1A**). Moreover, LINC00284 expression was upregulated in thyroid cancer samples collected in TCGA and GTEx databases (**Figure 1B**). In addition, the differential expression analysis of microarray data in the GSE97070 dataset indicated that miR-30d-5p was expressed at low levels in thyroid cancer (**Figure 1C**).

**Figure 1:** The expression of LINC00284 and miR-30d-5p in thyroid cancer tissues and cells. **(A)** LINC00284 expression in thyroid cancer in the GSE66783 microarray. **(B)** LINC00284 expression in thyroid cancer in the TCGA database; the abscissa represents the sample type, the ordinate represents the expression level, the red box indicates tumor samples, and the gray box indicates normal samples; *q < 0.01. **(C)** The GSE97070 microarray dataset showed that miR-30d-5p was downregulated in thyroid cancer. **(D)** The expression levels of LINC00284 and miR-30d-5p in HT-ori3, SW1736, FTC133, WRO82, HTh74, and C643 cell lines. *p < 0.05 compared with HT-ori3 cells. Data are presented as the means ± standard deviations, data were compared between two groups using unpaired *t-*test, and the experiments were repeated three times.

RETRACTED

RT-qPCR was then conducted to detect the patterns of LINC00284 and miR-30d-5p expression in thyroid cancer cells, and the subsequent results showed that the expression levels of LINC00284 were elevated in five thyroid cancer cell lines (SW1736, FTC133, WRO82, HTh74, and C643) relative to the normal thyroid epithelial cell line HT-ori3 (*p* < 0.05). In contrast, the levels of miR-30d-5p were noticeably lower in the five thyroid cancer cell lines (SW1736, FTC133, WRO82, HTh74, and C643) than in the normal thyroid epithelial cell line HT-ori3 (*p* < 0.05) (**Figure 1D**). Among the five thyroid cancer cell lines mentioned above, the HTh74 cell line exhibited the highest expression of LINC00284, while the C643 cell line showed the lowest expression levels of miR-30d-5p. Therefore, the HTh74 cell line and the C643 cell line were selected for subsequent cell transfection experiments.

### LINC00284 Silencing Inhibits the Malignant Biological Activities of Thyroid Cancer Cells

We genetically silenced LINC00284 in HTh74 cells by transfecting a LINC00284 shRNA to investigate the effect of LINC00284 on the biological activity of thyroid cancer cells. The RT-qPCR results indicated remarkably reduced expression levels of LINC00284 in HTh74 cells transfected with sh-LINC00284 compared with that of cells transfected with sh-NC (**Figure 2A**). Following the intervention, an MTT assay was performed to assess cell viability, and an ALDEFLUOR experiment was applied to detect the activity of ALDH, a stem cell-specific marker (20). Compared with cells transfected with sh-NC, the proliferation of HTh74 cells transfected with sh-LINC00284 was markedly suppressed at 48 and 72 h, while the proportion of cells with high ALDH activity was dramatically decreased (*p* < 0.05) (**Figures 2B, C**).

**Figure 2:** The effect of LINC00284 silencing on the malignant activities of thyroid cancer cells. **(A)** The expression of LINC00284 in HTh74 cells with different treatments was determined using RT-qPCR. **(B)** The viability of HTh74 cells with different treatments was determined using the MTT assay. **(C)** The ALDH activity of HTh74 cells with different treatments was determined using the ALDEFLUOR assay. **(D)** Flow cytometry analysis of the cell cycle of HTh74 cells with different treatments. **(E)** Apoptosis of HTh74 cells with different treatments was determined using flow cytometry. **(F)** The colony formation ability of HTh74 cells with different treatments. **(G)** Self-renewal ability of HTh74 cells with different treatments was assessed using cell sphere formation assay. **(H)** The invasive ability of HTh74 cells with different treatments was assessed using Transwell assay. *p < 0.05 compared with the cells transfected with sh-NC. Data are presented as the means ± standard deviations. Comparisons between two groups were analyzed using the unpaired *t*-test, and comparisons among groups at different time points were analyzed using repeated measurement ANOVA with Tukey’s *post hoc* test. The experiments were repeated three times.

RETRACTED

Moreover, the results of flow cytometry illustrated that LINC00284 silencing led to a higher percentage of apoptotic cells, an increased number of cells in G0/G1 phase, and a decreased number of cells in the S phase (*p* < 0.05) (**Figures 2D, E**). Based on the results of colony formation, cell sphere formation, and Transwell assays, the numbers of colonies, cell spheres, and invasive HTh74 cells were substantially decreased after LINC00284 knockdown (*p* < 0.05) (**Figures 2F–H**). Together, the abovementioned results indicated that LINC00284 silencing suppressed HTh74 cell proliferation, viability, colony formation, and invasion abilities and promoted apoptosis.

### LINC00284 Upregulates ADAM12 by Competitively Binding to miR-30d-5p

Prediction results from the bioinformatics website lncLocator indicated that LINC00284 was primarily located in the cytoplasm (**Figure 3A**). Furthermore, the FISH assay and RT-qPCR validated that LINC00284 was mainly located in the cytoplasm of HTh74 cells (**Figures 3B, C**). Moreover, the results of the miRDB website analysis revealed the presence of a specific binding region between LINC00284 and miR-30d-5p (**Figure 3D**). In addition, the results of the dual-luciferase reporter gene assay showed that the luciferase activity of the LINC00284-WT plasmid was noticeably reduced after cotransfection with the miR-30d-5p mimic (*p* < 0.05), but no significant differences were noted in the cell groups transfected with the LINC00284-MUT plasmid (*p* > 0.05) (**Figure 3E**).

**Figure 3:** The regulatory relationship among LINC00284, miR-30d-5p, and ADAM12. **(A)** The localization of LINC00284 in cells predicted by a bioinformatics website. **(B)** The localization of LINC00284 in HTh74 cells detected using the FISH assay. **(C)** The localization of LINC00284 in HTh74 cells detected using RT-qPCR, * *p* < 0.05 compared with the cytoplasm. **(D)** The binding sites for LINC00284 and miR-30d-5p analyzed using the miRDB website. **(E)** The binding relationship between LINC00284 and miR-30d-5p was identified by conducting a dual-luciferase reporter assay, *p < 0.05 compared with cells transfected with the NC mimic. **(F)** The relationship between LINC00284 and miR-30d-5p was detected using an RNA pull-down assay, *p < 0.05 compared with cells transfected with Bio-NC or Bio-LINC00284-MUT. **(G)** The binding of LINC00284 to the AGO2 protein was detected using a RIP assay, *p < 0.05 compared with cells binding to IgG. **(H)** The binding sites for miR-30d-5p and ADAM12 predicted by the TargetScan website. **(I)** ADAM12 expression in thyroid cancer samples in the TCGA database; the red box indicates tumor samples, and the purple box indicates normal samples (FDR = 1.1e-7). **(J)** Correlation analysis of miR-30d-5p and ADAM12 expression in the TCGA database. The correlation coefficient and correlation *p* value are shown in the upper left of the panel. **(K)** The binding relationship between miR-30d-5p and ADAM12 was verified by dual-luciferase reporter assay, *p < 0.05 compared with cells transfected with the NC mimic. **(L)** Western blot analysis of ADAM12 protein expression in C643 thyroid cancer cells after the overexpression of LINC00284 or miR-30d-5p. *p < 0.05 compared with cells transfected with oe-NC, ^#^ *p* < 0.05 compared with cells transfected with the miR-30d-5p mimic, ^&^ *p* < 0.05 compared with cells transfected with oe-LINC00284 + NC mimic. Data are presented as the means ± standard deviations. Comparisons between two groups were analyzed using unpaired *t*-tests, and comparisons among multiple groups were analyzed using one-way ANOVA, followed by Tukey’s *post hoc* test. The experiments were repeated three times.

RETRACTED

We performed a biotin-labeled RNA pull-down experiment to further verify whether miR-30d-5p is enriched and regulated by LINC00284. Compared with the samples subjected to pull-down with Bio-NC and Bio-LINC00284-MUT, miR-30d-5p was enriched in the samples pulled down by Bio-LINC00284-WT (*p* < 0.05) (**Figure 3F**). LncRNAs are widely reported to be able to serve as molecular sponges or ceRNAs that regulate the aggregation and biological function of miRNAs (21). Subsequently, a RIP assay was performed to identify the binding of LINC00284 to the AGO2 protein. Compared with the IgG group, the binding of LINC00284 to AGO2 protein was noticeably enhanced (**Figure 3G**). These findings collectively indicated that LINC00284 competitively bound to miR-30d-5p.

Furthermore, the prediction results of TargetScan suggested that ADAM12 might be a target gene of miR-30d-5p (**Figure 3H**). Subsequently, the expression patterns of ADAM12 in thyroid cancer samples in the TCGA database were retrieved, which revealed high expression of ADAM12 in thyroid cancer (**Figure 3I**). Moreover, the correlation analysis indicated a significant negative correlation between miR-30d-5p and ADAM12 expression (**Figure 3J**), which further suggested that ADAM12 may be directly regulated by miR-30d-5p. A dual-luciferase reporter assay was performed to further verify this relationship, and the luciferase activity of cells transfected with ADAM12-WT decreased dramatically after cotransfection with the miR-30d-5p mimic, while the luciferase activity was unaffected in the cell groups transfected with ADAM12-MUT (**Figure 3K**).

RETRACTED

Additionally, the expression patterns of the ADAM12 protein in C643 cells overexpressing LINC00284 or miR-30d-5p were determined using Western blot analysis. Levels of the ADAM12 protein were dramatically increased following LINC00284 overexpression but were reduced after the overexpression of miR-30d-5p; moreover, overexpression of miR-30d-5p reversed the effect of LINC00284 overexpression on promoting ADAM12 protein expression (**Figure 3L**). In summary, the aforementioned results support the hypothesis that LINC00284 competitively bound to miR-30d-5p and subsequently upregulated the expression of ADAM12.

### LINC00284 Enhances the Malignant Biological Activities of Thyroid Cancer Cells by Impairing miR-30d-5p-Dependent Inhibition of ADAM12

C643 cells were transfected with the miR-30d-5p mimic, oe-LINC00284, and oe-ADAM12 alone or in combination to analyze the effects of LINC00284/miR-30d-5p/ADAM12 on thyroid cancer cells. The patterns of LINC00284, miR-30d-5p, and ADAM12 expression were subsequently measured using RT-qPCR, and the results showed that miR-30d-5p overexpression did not alter the expression of LINC00284 in C643 cells but dramatically reduced the expression of the ADAM12 mRNA. However, the expression levels of ADAM12 mRNA were upregulated, while the expression of miR-30d-5p was decreased in C643 cells cotransfected with the miR-30d-5p mimic and oe-LINC00284 compared to C643 cells cotransfected with the miR-30d-5p mimic and oe-NC. Additionally, cotransfection with the miR-30d-5p mimic and oe-ADAM12 significantly increased the expression of the ADAM12 mRNA without affecting LINC00284 and miR-30d-5p expression compared to cotransfection with the miR-30d-5p mimic and oe-NC (**Figure 4A**).

**Figure 4:** The effect of the LINC00284/miR-30d-5p/ADAM12 axis on the biological activity of thyroid cancer cells. **(A)** The expression of LINC00284, miR-30d-5p and ADAM12 mRNA in C643 cells was determined using RT-qPCR. **(B)** The viability of C643 cells was determined using the MTT assay. **(C)** The ALDH activity of C643 cells was determined using the ALDEFLUOR experiment. **(D)** Flow cytometry analysis of the cell cycle of C643 cells d. **(E)** The apoptosis of C643 cells was determined using flow cytometry. **(F)** The colony formation ability of C643 cells. **(G)** Self-renewal ability of C643 cells assessed using the cell sphere formation assay. **(H)** The invasive ability of C643 cells assessed using the Transwell assay. *p < 0.05 compared with cells transfected with sh-NC. Data are presented as the means ± standard deviations. Comparisons between two groups were analyzed using the unpaired *t*-test, comparisons among multiple groups were analyzed using one-way ANOVA, followed by Tukey’s *post hoc* test, and comparisons among groups at different time points were analyzed using repeated measures ANOVA with Tukey’s *post hoc* test. The experiments were repeated 3 times. ^#^ *p* < 0.05 compared with cells transfected with miR-30d-5p mimic + oe-NC.

RETRACTED

Afterwards, changes in the biological activity of transfected C643 cells were assessed accordingly. Transfection of the miR-30d-5p mimic induced noticeable reductions in the viability of C643 cells and proportion of cells with high ALDH activity (**Figures 4B, C**), increased the number of cells in the G0/G1 phase and decreased the number of cells in the S phase (**Figure 4D**), accelerated cell apoptosis (**Figure 4E**), and decreased the numbers of colonies (**Figure 4F**), cell spheres (**Figure 4G**), and invasive cells (**Figure 4H**). However, these effects of the miR-30d-5p mimic were reversed by transfection of oe-LINC00284 or oe-ADAM12 (**Figures 4B–H**). In summary, overexpression of miR-30d-5p inhibited the proliferative and invasive potential of C643 cells while promoting their apoptosis. Additionally, overexpression of LINC00284 or ADAM12 reversed the effect of miR-30d-5p overexpression on the biological activities of C643 cells.

### LINC00284 Activates the Notch Signaling Pathway by Competitively Binding to miR-30d-5p to Increase ADAM12 Expression

The Notch signaling pathway is known to play an important role in regulating cell growth and apoptosis and is activated in various types of thyroid cancer (22–24). Western blot analysis was performed to detect the expression patterns of Notch pathway-related proteins in HTh74 cells with LINC00284 knockdown to explore the specific mechanism by which LINC00284 competitively binds to miR-30d-5p in thyroid cancer cells. Levels of both the Notch1 and HES1 proteins were reduced in HTh74 cells transfected with sh-LINC00284 (**Figure 5A**).

**Figure 5:** The effect of the competitive binding of LINC00284 to miR-30d-5p to regulate the ADAM12/Notch axis on the biological activity of thyroid cancer cells. LINC00284 competitively binds to miR-30d-5p to upregulate the expression of ADAM12 and activate the Notch signaling pathway. **(A)** The expression of Notch1 and HES1 proteins in HTh74 cells was measured using Western blot analysis, *p < 0.05 compared with cells transfected with sh-NC. **(B)** The expression of Notch1 and HES1 proteins in C643 cells was measured using Western blot analysis, *p < 0.05 compared with cells transfected with sh-NC or NC mimic, ^#^ *p* < 0.05 compared with cells transfected with miR-30d-5p mimic + oe-NC. **(C)** The expression of Notch1 and HES1 proteins in HTh74 cells was measured using Western blot analysis. **(D)** The viability of HTh74 cells was determined using the MTT assay. **(E)** The ALDH activity of HTh74 cells determined in the ALDEFLUOR experiment. **(F)** Flow cytometry analysis of the cell cycle of HTh74 cells. **(G)** Flow cytometry analysis of the apoptosis of HTh74 cells. **(H)** The colony formation ability of C643 cells. **(I)** Self-renewal ability of C643 cells assessed using the cell sphere formation assay. **(J)** The invasive ability of C643 cells assessed using the Transwell assay. *p < 0.05 compared with cells treated with sh-LINC00284 + DMSO. Measurement data are presented as the means ± standard deviations. Comparisons between two groups were analyzed using the unpaired *t*-test, comparisons among multiple groups were analyzed using one-way ANOVA followed by Tukey’s *post hoc* test, and comparisons among groups at different time points were analyzed using repeated measures ANOVA with Tukey’s *post hoc* test. The experiments were repeated three times.

RETRACTED

Next, C643 cells were separately transfected with miR-30d-5p mimic, oe-LINC00284, and oe-ADAM12 alone or in combination. The results of Western blot analyses illustrated dramatically reduced levels of the Notch1 and HES1 proteins in C643 cells transfected with the miR-30d-5p mimic, while these effects were negated by the transfection of oe-LINC00284 or oe-ADAM12 (**Figure 5B**). These findings supported the hypothesis that the upregulation of LINC00284 regulated the expression of ADAM12 by competitively binding to miR-30d-5p, thereby activating the Notch signaling pathway.

HTh74 cells were treated with the ERK signaling pathway activator TBHQ after transfection with sh-LINC00284. TBHQ treatment reversed the reduction in the expression of the Notch1 and HES1 proteins caused by LINC00284 silencing (**Figure 5C**). In addition, the biological activities of HTh74 cells were assessed after sh-LINC00284 transfection or TBHQ treatment, and compared with cells treated with sh-LINC00284 + DMSO, the viability of HTh74 cells and the proportion of cells with high ALDH activity were reduced, apoptosis was accelerated, the number of cells in the G0/G1 phase was increased, the number of cells in the S phase was decreased, and colony formation, sphere formation, and cell invasion were all suppressed following treatment with sh-LINC00284 + TBHQ (*p* < 0.05) (**Figures 5D–J**). Based on these results, LINC00284 activated the Notch signaling pathway and subsequently regulated the biological activity of thyroid cancer cells through the miR-30d-5p/ADAM12 axis.

RETRACTED

### LINC00284 Enhances the Tumorigenic Ability of Thyroid Cancer Cells by Repressing miR-30d-5p

The tumorigenesis ability of thyroid cancer cells was tested by establishing xenograft tumors in nude mice. The results presented in **Figures 6A–C** illustrated that compared with the oe-NC group, the volume and weight of tumors were dramatically increased in nude mice from the oe-LINC00284 group but were significantly reduced in the LV-miR-30d-5p group compared to the LV-NC group. Additionally, miR-30d-5p reversed the effects of LINC00284 on the volume and weight of tumors in nude mice.

**Figure 6:** The effect of LINC00284-mediated miR-30d-5p silencing on the tumorigenic ability of thyroid cancer cells. **(A)** Representative pictures of xenograft tumors in nude mice. **(B)** Statistical analysis of the tumor volume in nude mice. **(C)** Statistical analysis of the tumor weight in nude mice. **(D)** The expression of LINC00284, miR-30d-5p, and ADAM12 mRNA in tumor tissues was determined using RT-qPCR. **(E)** The expression of ADAM12 in tumor tissues measured using Western blot analysis. *p < 0.05 compared with mice injected with oe-NC-infected cancer cells, ^#^ *p* < 0.05 compared with mice injected with LV-NC-infected cancer cells, and ^&^ *p* < 0.05 compared with mice injected with oe-LINC00284+ LV-NC-infected cancer cells. Data are presented as the means ± standard deviations. Comparisons between two groups were analyzed using the unpaired *t*-test, comparisons among multiple groups were analyzed using one-way ANOVA followed by Tukey’s *post hoc* test, and comparisons among groups at different time points were analyzed using repeated measures ANOVA with Tukey’s *post hoc* test. The experiments were repeated three times.

RT-qPCR and Western blot analyses were then conducted to detect the expression patterns of LINC00284, miR-30d-5p, and ADAM12 in tumor tissues. Compared with mice transfected with oe-NC, the expression levels of LINC00284 and ADAM12 increased, and the expression levels of miR-30d-5p were obviously decreased in tumor tissues from nude mice following the injection of cells transfected with oe-LINC00284. Compared with tumor cells transfected with LV-NC, no significant differences in the expression levels of LINC00284 were observed, whereas the expression of miR-30d-5p increased, and the expression of ADAM12 decreased in tumor tissues from nude mice injected with cells transfected with LV-miR-30d-5p. Compared with tumor cells transfected with oe-LINC00284 + LV-NC, no significant differences in LINC00284 expression levels were observed, while the expression levels of miR-30d-5p were upregulated and the expression levels of ADAM12 were downregulated in tumor tissues from nude mice injected with cells cotransfected with oe-LINC00284+ LV-miR-30d-5p (**Figures 6D, E**). In conclusion, these findings indicated that overexpression of LINC00284 promoted thyroid tumorigenesis in thyroid cancer, while miR-30d-5p overexpression inhibited tumorigenesis. Moreover, overexpression of miR-30d-5p inhibited tumorigenesis induced by LINC00284 overexpression.

RETRACTED

## Discussion

Thyroid cancer stems from follicular or parafollicular thyroid cells and its incidence rates have increased; despite efficacious treatment, it still presents with abysmal 5 year survival rates (25). LncRNAs, which function as ceRNAs of miRNAs, possess the ability to regulate the expression of RNA targets through miRNA response elements, whereas a few studies have also highlighted the presence of some ceRNA regulatory mechanisms in thyroid cancer (26). Expanding on our current knowledge, the findings obtained in our study indicated that the downregulation of LINC00284 suppressed proliferation and invasion while promoting the apoptosis of thyroid cancer cells through the miR-30d-5p-dependent inhibition of ADAM12 expression and blockade of the Notch signaling pathway.

First, our data revealed that LINC00284 was expressed at high levels in thyroid cancer. Interestingly, LINC00284 expression levels have previously been reported to be associated with the overall survival of patients with PTC, another malignancy of the thyroid (26). Another study documented the upregulation of LINC00284 in ovarian cancer, and its high expression levels were associated with poor outcomes in patients (27). Accordingly, a plausible hypothesis would be that LINC00284 plays a crucial role in the progression and outcomes of thyroid cancer and might serve as a promising therapeutic target for this malignancy. Furthermore, our findings revealed low expression of miR-30d-5p in thyroid cancer. Notably, the downregulation of miR-30d was previously reported in human anaplastic thyroid carcinoma (ATC) and further contributed to cancer development (15). In addition, Zhang et al. highlighted that the dysregulation of miR-30d affects the autophagy-mediated survival of human ATC cells and has been regarded as a potential target for the treatment of ATC (28). Moreover, a number of studies have indicated the role of miR-30d-5p as a tumor suppressor in diverse human cancers. For instance, overexpression of miR-30d-5p inhibits prostate cancer cell proliferation and invasion while promoting cell apoptosis (16). In gallbladder carcinoma, miR-30d-5p was also documented to be expressed at low levels, while its overexpression suppressed cancer progression (29, 30). Therefore, in addition to LINC00284, miR-30d plays a role in the fate of thyroid cancer and warrants further investigation.

RETRACTED

Most recently, lncRNAs have emerged as important factors that are capable of diminishing miRNA activity by competitively binding to miRNAs through common miRNA response elements, where lncRNAs promote the expression of target RNAs (31). In addition, an integrated analysis has suggested the presence of a LINC00284-associated ceRNA network in gastric cancer, hence underscoring potential targets for the treatment of gastric cancer (32). In accordance with the abovementioned data, our experimental findings indicated that LINC00284 competitively bound to miR-30d-5p and inhibited its expression, suggesting the participation of the LINC00284-miR-30d-5p regulatory network in the development of thyroid cancer.

Furthermore, during the course of our study, we identified ADAM12 as the target gene of miR-30d-5p. Inherently, ADAM12 is known to play a role in cell proliferation. More interestingly, hsa-miR-145-3p, hsa-miR-145-5p, and hsa-miR-490-3p are downregulated, whereas their target genes, including ADAM12, ACAN, HOXC11, and MMP11, are upregulated in cancer cells (33). In addition, ADAM12 belongs to the disintegrin and metalloproteinase family that has been previously documented to be abnormally expressed and thus associated with the pathogenesis of numerous malignancies (34). For instance, ADAM12 is expressed at aberrantly high levels in esophageal cancer tissues, while its suppression inhibits cancer development (35). During our study, we elucidated that LINC00284 silencing or miR-30d-5p overexpression attenuated the malignant biological activities of thyroid cancer cells. However, LINC00284 or ADAM12 overexpression reversed the effects of miR-30d-5p on thyroid cancer cells. Altogether, our findings indicated that LINC00284 bound to miR-30d-5p and upregulate ADAM12 expression, thus serving as a promoter of thyroid cancer progression.

Finally, our experimental findings also showed that LINC00284 activated the Notch signaling pathway by increasing ADAM12 expression. The aforementioned activation of the Notch signaling pathway has also been previously implicated in the progression of PTC (36). The Notch pathway directly combines events at the cell membrane with transcriptional regulation. The sequential proteolytic cleavage of the Notch receptor may release the signal-transducing Notch intracellular domain (NICD) into the cytoplasm that subsequently enters the nucleus to bind to the CBF-1/Su(H)/LAG1 (CSL) transcription factor to form a NICD/CSL transcription activation complex. This complex further activates transcriptional regulators of the basic-helix-loop-helix (bHLH) class that primarily act as repressors, such as HES, HEY, and HERP, which play important biological roles in tumors (37). The Notch signaling pathway is present in normal adult thyrocytes and is modulated by thyroid-stimulating hormone (38). The Notch signaling pathway has been reported to play various roles in diverse tissues and organisms to determine cell fate, and it also functions as a critical factor regulating stem cell self-renewal (39). Aberrantly activated Notch signaling enhances the malignant behaviors of thyroid cancer cells (40). Inhibition of this pathway has also been noted to limit the progression of thyroid cancer (23). Furthermore, ADAM family members serve as crucial factors in the Notch signaling pathway; for example, ADAM17 is indispensable for Notch signaling pathway activation (41). Based on our results, LINC00284 induced the activation of the Notch signaling pathway by increasing ADAM17 expression, thereby promoting thyroid cancer development.

RETRACTED

In summary, our study provides evidence that LINC00284 may competitively bind to miR-30d-5p to increase ADAM12 expression in thyroid cancer cells, which further induces the activation of the Notch signaling pathway and subsequently promotes the growth and invasion while inhibiting the apoptosis of thyroid cancer cells (**Figure 7**). Thus, LINC00284 is suggested to participate in a network that potentially regulates the development of thyroid cancer. Future efforts and clinical data are expected to validate our findings and facilitate the development of efficacious therapeutic targets for thyroid cancer.

**Figure 7:** Schematic diagram of the molecular mechanism showing that LINC00284 competitively binds to miR-30d-5p to regulate ADAM12 expression, thus participating in the development of thyroid cancer through the Notch signaling pathway.

## Data Availability Statement

The original contributions presented in the study are included in the article/**Supplementary Material**. Further inquiries can be directed to the corresponding author.

## Ethics Statement

The animal study was reviewed and approved by the Second Hospital of Jilin University.

## Author Contributions

RQ and CH designed the study. ZK and LG collated the data, carried out data analyses, and produced the initial draft of the manuscript. RQ and FQ contributed to drafting the manuscript. All authors have read and approved the final submitted manuscript.

RETRACTED

## Funding

This study was supported by the Science and Technology Department of Jilin Province, P.R.C. [grant number 20200201543JC].

## Conflict of Interest

The authors declare that the research was conducted in the absence of any commercial or financial relationships that could be construed as a potential conflict of interest.

## References

[1] CabanillasMEMcFaddenDGDuranteC. Thyroid Cancer. Lancet (2016) 388:2783–95. 10.1016/S0140-6736(16)30172-6 27240885

[2] RomanBRMorrisLGDaviesL. The Thyroid Cancer Epidemic, 2017 Perspective. Curr Opin Endocrinol Diabetes Obes (2017) 24:332–6. 10.1097/MED.0000000000000359 PMC586411028692457

[3] ChmielikERusinekDOczko-WojciechowskaMJarzabMKrajewskaJCzarnieckaA. Heterogeneity of Thyroid Cancer. Pathobiology (2018) 85:117–29. 10.1159/000486422 29408820

[4] MuGWangHCaiZJiH. OPN -443C>T Genetic Polymorphism and Tumor OPN Expression Are Associated With the Risk and Clinical Features of Papillary Thyroid Cancer in a Chinese Cohort. Cell Physiol Biochem (2013) 32:171–9. 10.1159/000350133 23867349

[5] DengXWuBXiaoKKangJXieJZhangX. MiR-146b-5p Promotes Metastasis and Induces Epithelial-Mesenchymal Transition in Thyroid Cancer by Targeting ZNRF3. Cell Physiol Biochem (2015) 35:71–82. 10.1159/000369676 25547151

[6] LiQLiHZhangLZhangCYanWWangC. Identification of Novel Long Non-Coding RNA Biomarkers for Prognosis Prediction of Papillary Thyroid Cancer. Oncotarget (2017) 8:46136–44. 10.18632/oncotarget.17556 PMC554225528545026

[7] QiuZLShenCTSunZKWeiWJZhangXYSongHJ. Circulating Long Non-Coding RNAs Act as Biomarkers for Predicting 131i Uptake and Mortality in Papillary Thyroid Cancer Patients With Lung Metastases. Cell Physiol Biochem (2016) 40:1377–90. 10.1159/000453190 27997908

[8] TengHMaoFLiangJXueMWeiWLiX. Transcriptomic Signature Associated With Carcinogenesis and Aggressiveness of Papillary Thyroid Carcinoma. Theranostics (2018) 8:4345–58. 10.7150/thno.26862 PMC613493630214625

[9] LiGKongQ. LncRNA LINC00460 Promotes the Papillary Thyroid Cancer Progression by Regulating the LINC00460/miR-485-5p/Raf1 Axis. Biol Res (2019) 52:61. 10.1186/s40659-019-0269-9 31870440PMC6929379

[10] RuanZZhaoD. Long Intergenic Noncoding RNA LINC00284 Knockdown Reduces Angiogenesis in Ovarian Cancer Cells Via Up-Regulation of MEST Through NF-KappaB1. FASEB J (2019) 33:12047–59. 10.1096/fj.201900101RR PMC690273131574234

[11] FanMLiXJiangWHuangYLiJWangZ. A Long Non-Coding RNA, PTCSC3, as a Tumor Suppressor and a Target of miRNAs in Thyroid Cancer Cells. Exp Ther Med (2013) 5:1143–6. 10.3892/etm.2013.933 PMC362871823599737

[12] YangXZChengTTHeQJLeiZYChiJTangZ. LINC01133 as ceRNA Inhibits Gastric Cancer Progression by Sponging miR-106a-3p to Regulate APC Expression and the Wnt/Beta-Catenin Pathway. Mol Cancer (2018) 17:126. 10.1186/s12943-018-0874-1 30134915PMC6106894

RETRACTED

[13] ChouCKChenRFChouFFChangHWChenYJLeeYF. miR-146b is Highly Expressed in Adult Papillary Thyroid Carcinomas With High Risk Features Including Extrathyroidal Invasion and the BRAF(V600E) Mutation. Thyroid (2010) 20:489–94. 10.1089/thy.2009.0027 20406109

[14] BoufraqechMZhangLJainMPatelDEllisRXiongY. miR-145 Suppresses Thyroid Cancer Growth and Metastasis and Targets AKT3. Endocr Relat Cancer (2014) 21:517–31. 10.1530/ERC-14-0077 PMC837557124781864

[15] EspositoFTornincasaMPallantePFedericoABorboneEPierantoniGM. Down-Regulation of the miR-25 and miR-30d Contributes to the Development of Anaplastic Thyroid Carcinoma Targeting the Polycomb Protein EZH2. J Clin Endocrinol Metab (2012) 97:E710–8. 10.1210/jc.2011-3068 22399519

[16] SongYSongCYangS. Tumor-Suppressive Function of miR-30d-5p in Prostate Cancer Cell Proliferation and Migration by Targeting NT5E. Cancer Biother Radiopharm (2018) 33:203–11. 10.1089/cbr.2018.2457 29916747

[17] RaoVHVogelKYanagidaJKMarwahaNKandelATrempusC. Erbb2 Up-Regulation of ADAM12 Expression Accelerates Skin Cancer Progression. Mol Carcinog (2015) 54:1026–36. 10.1002/mc.22171 24798404

[18] DiazBYuenAIizukaSHigashiyamaSCourtneidgeSA. Notch Increases the Shedding of HB-EGF by ADAM12 to Potentiate Invadopodia Formation in Hypoxia. J Cell Biol (2013) 201:279–92. 10.1083/jcb.201209151 PMC362851723589494

[19] RobinsonMDMcCarthyDJSmythGK. edgeR: A Bioconductor Package for Differential Expression Analysis of Digital Gene Expression Data. Bioinformatics (2010) 26:139–40. 10.1093/bioinformatics/btp616 PMC279681819910308

[20] LiangDShiY. Aldehyde Dehydrogenase-1 Is a Specific Marker for Stem Cells in Human Lung Adenocarcinoma. Med Oncol (2012) 29:633–9. 10.1007/s12032-011-9933-9 21484084

[21] KarrethFAPandolfiPP. ceRNA Cross-Talk in Cancer: When Ce-Bling Rivalries Go Awry. Cancer Discov (2013) 3:1113–21. 10.1158/2159-8290.CD-13-0202 PMC380130024072616

[22] GreenblattDYCayoMAAdlerJTNingLHaymartMRKunnimalaiyaanM. Valproic Acid Activates Notch1 Signaling and Induces Apoptosis in Medullary Thyroid Cancer Cells. Ann Surg (2008) 247:1036–40. 10.1097/SLA.0b013e3181758d0e PMC290480918520232

[23] WanJFWanJYDongCLiL. Linc00324 Promotes the Progression of Papillary Thyroid Cancer Via Regulating Notch Signaling Pathway. Eur Rev Med Pharmacol Sci (2020) 24:6818–24. 10.26355/eurrev_202006_21671 32633374

[24] GalloCFragliassoVDonatiBTorricelliFTameniAPianaS. The bHLH Transcription Factor DEC1 Promotes Thyroid Cancer Aggressiveness by the Interplay With NOTCH1. Cell Death Dis (2018) 9:871. 10.1038/s41419-018-0933-y 30158530PMC6115386

RETRACTED

[25] ZhaoJJHaoSWangLLHuCYZhangSGuoLJ. Long Non-Coding RNA ANRIL Promotes the Invasion and Metastasis of Thyroid Cancer Cells Through TGF-Beta/Smad Signaling Pathway. Oncotarget (2016) 7:57903–18. 10.18632/oncotarget.11087 PMC529539927507052

[26] ZhaoYWangHWuCYanMWuHWangJ. Construction and Investigation of lncRNA-Associated ceRNA Regulatory Network in Papillary Thyroid Cancer. Oncol Rep (2018) 39:1197–206. 10.3892/or.2018.6207 PMC580203429328463

[27] WangLPengQSaiBZhengLXuJYinN. Ligand-Independent EphB1 Signaling Mediates TGF-Beta-Activated CDH2 and Promotes Lung Cancer Cell Invasion and Migration. J Cancer (2020) 11:4123–31. 10.7150/jca.44576 PMC719625632368295

[28] ZhangYYangWQZhuHQianYYZhouLRenYJ. Regulation of Autophagy by miR-30d Impacts Sensitivity of Anaplastic Thyroid Carcinoma to Cisplatin. Biochem Pharmacol (2014) 87:562–70. 10.1016/j.bcp.2013.12.004 PMC392620124345332

[29] HeYChenXYuYLiJHuQXueC. LDHA is a Direct Target of miR-30d-5p and Contributes to Aggressive Progression of Gallbladder Carcinoma. Mol Carcinog (2018) 57:772–83. 10.1002/mc.22799 29569755

[30] LiuKXuQ. LncRNA PVT1 Regulates Gallbladder Cancer Progression Through miR-30d-5p. J Biol Regul Homeost Agents (2020) 34:875–83. 10.23812/20-180-A-32 32689767

[31] SalmenaLPolisenoLTayYKatsLPandolfiPP. A ceRNA Hypothesis: The Rosetta Stone of a Hidden RNA Language? Cell (2011) 146:353–8. 10.1016/j.cell.2011.07.014 PMC323591921802130

[32] XingCCaiZGongJZhouJXuJGuoF. Identification of Potential Biomarkers Involved in Gastric Cancer Through Integrated Analysis of Non-Coding RNA Associated Competing Endogenous RNAs Network. Clin Lab (2018) 64:1661–9. 10.7754/Clin.Lab.2018.180419 30336538

[33] LiuJLiuFShiYTanHZhouL. Identification of Key miRNAs and Genes Associated With Stomach Adenocarcinoma From The Cancer Genome Atlas Database. FEBS Open Bio (2018) 8:279–94. 10.1002/2211-5463.12365 PMC579447129435418

[34] YinHZhongFOuyangYWangQDingLHeS. Upregulation of ADAM12 Contributes to Accelerated Cell Proliferation and Cell Adhesion-Mediated Drug Resistance (CAM-DR) in Non-Hodgkin’s Lymphoma. Hematology (2017) 22:527–35. 10.1080/10245332.2017.1312205 28395594

[35] LuoMLZhouZSunLYuLSunLLiuJ. An ADAM12 and FAK Positive Feedback Loop Amplifies the Interaction Signal of Tumor Cells With Extracellular Matrix to Promote Esophageal Cancer Metastasis. Cancer Lett (2018) 422:118–28. 10.1016/j.canlet.2018.02.031 29476791

[36] YeYSongYZhuangJHeSNiJXiaW. Long Noncoding RNA CCAL Promotes Papillary Thyroid Cancer Progression by Activation of NOTCH1 Pathway. Oncol Res (2018) 26:1383–90. 10.3727/096504018X15188340975709 PMC784464929471887

RETRACTED

[37] MeuretteOMehlenP. Notch Signaling in the Tumor Microenvironment. Cancer Cell (2018) 34:536–48. 10.1016/j.ccell.2018.07.009 30146333

[38] GuoZHardinHLloydRV. Cancer Stem-Like Cells and Thyroid Cancer. Endocr Relat Cancer (2014) 21:T285–300. 10.1530/ERC-14-0002 24788702

[39] LiuJSatoCCerlettiMWagersA. Notch Signaling in the Regulation of Stem Cell Self-Renewal and Differentiation. Curr Top Dev Biol (2010) 92:367–409. 10.1016/S0070-2153(10)92012-7 20816402

[40] ChoiDRamuSParkEJungEYangSJungW. Aberrant Activation of Notch Signaling Inhibits Prox1 Activity to Enhance the Malignant Behavior of Thyroid Cancer Cells. Cancer Res (2016) 76:582–93. 10.1158/0008-5472.CAN-15-1199 PMC473816026609053

[41] ChristianLM. The ADAM Family: Insights Into Notch Proteolysis. Fly (Austin) (2012) 6:30–4. 10.4161/fly.18823 22513479

